The article "A Study on Course of Infection and Haematological Changes in falciparum-Infected in Comparison with Artemisinin(s)-Treated Mice" was retracted in 2014. Reasons: errors in the data; errors in the results or conclusions; concerns about the data; concerns about the results or conclusions.

# A Study on Course of Infection and Haematological Changes in *falciparum*-Infected in Comparison with Artemisinin(s)-Treated Mice

**DOI:** 10.1155/2013/426040

**Published:** 2013-06-11

**Authors:** Kalyan Kumar Kuthala, Sowjanya Meka, Sunita Kanikaram

**Affiliations:** Department of Zoology and Aquaculture, Acharya Nagarjuna University, Nagarjunanagar, Guntur, Andhra Pradesh 522 510, India

## Abstract

To find out the efficacy and effect of artemisinin derivatives on haematological indices, C57BL/6J mice were challenged with *Plasmodium falciparum* and treated with therapeutic doses of AS, AE, and AL. Course of infection was studied in the infected and treated groups up to day 42. Peak level of parasitaemia (38%) was observed on day 11 in infected group. Haematological indices indicated significant (*P* < 0.05) decrease in RBC, WBC, haemoglobin, packed cell volume, mean cell volume, and platelet counts in infected mice. But all the parameters were restored to normal values, and significant (*P* < 0.05) changes were observed in all drug-treated groups. Insignificant changes were observed for MCHC (*P* > 0.05) in all drug-treated groups. Percent of peak parasitaemia was much reduced in AL- (3.2% on day 3) treated group in comparison with AE- (2.4% on day 4) and AS- (4% on day 2) treated groups. Parasites were completely cleared on day 6 in AS group, day 5 in AE group, and day 4 in AL group. Hence, our results strongly support that combination therapy has high efficacy rates than monotherapy. No adverse effects were observed on haematological parameters when animals were treated with therapeutic dosages.

## 1. Introduction

Despite advances in knowledge, malaria continues to cause significant morbidity and mortality worldwide. Over 40% of the world population lives in malaria-endemic areas and it is very high (20%) in severe malaria (parasitaemia > 5%). Today malaria is the most important problem for which an estimated 300–500 million cases were recorded and 1.5–2.7 million deaths occur each year [1]. Among them 19,500 death cases due to malaria have been recorded in India [2]. Mortality rate usually depends on the management of malaria which involves antimalarial drug resistance of *Plasmodium falciparum* and occurrence of systemic complications. Most of the systemic complications from malaria are mainly because of hyperparasitaemia [3].

Blood is the most easily accessible diagnostic tissue. Variations in haematological parameters are influenced by any disease condition which affects the haemopoietic physiology. This is likely to happen with an endemic disease such as malaria that affects the host homeostasis [4]. The target of malaria parasite is RBC so that peripheral blood smear examination is the major diagnostic tool of the disease. Microscopic diagnosis is the “imperfect gold standard” for malaria parasite detection and species identification. This technique requires technical expertise and time consuming in repeated smear examinations [5]. However, it is a valuable technique when performed correctly in the right hands but can be unreliable and perceived as useless when poorly executed [6, 7].

The article "A Study on Course of Infection and Haematological Changes in falciparum-Infected in Comparison with Artemisinin(s)-Treated Mice" was retracted in 2014. Reasons: errors in the data; errors in the results or conclusions; concerns about the data; concerns about the results or conclusions.

Haematological changes associated with malaria infection are well recognized, but specific changes may differ from the level of malaria endemicity, background haemoglobinopathy, nutritional status, demographic factors, and immunity to malaria [8]. Hence, haematological changes are the most common and important complications encountered and are considered a hallmark of malaria, playing a major role in the fatality. Prediction of the haematological changes enables the clinician to establish an effective and early therapeutic intervention in order to prevent the occurrence of major complications [3]. The haematological abnormalities that have been reported include anaemia, thrombocytopenia, lymphocytosis and rarely disseminated intravascular coagulation [9], leucopenia, leucocytosis, neutropenia, neutrophilia, and eosinophilia, and monocytosis also have been reported [10, 11]. 

Artemisinin(s) monotherapy and combination therapy (ACTs) are currently used as first line treatment for uncomplicated malaria. Artesunate is a semisynthetic derivative of artemisinin consisting of sodium succinyl salt of dihydroartemisinin, a potent blood schizonticide highly effective against multidrug resistant strains of *P. falciparum*. Hence it is widely used for the treatment of malaria [12]. *α*, β arteether (30 : 70 mixture of enantiomers) is a fast-acting blood schizonticide completed multicentric clinical trials in *P. falciparum* endemic areas and was found to be effective and marketed in 1997 as E Mal. Arteether has a higher safety margin compared to other artemisinin derivatives, has longer half-life, and produces high cure rates when administered in a short 3-dose (*i.m.*) regimen [13]. Artemether + lumefantrine combination combines the benefits of a rapid short-lived schizonticidal effect of arteether with a slower but longer acting schizonticidal effect of Lumefantrine, a highly lipophilic aryl amino alcohol.

The present study was aimed to reveal the effect of 3 frequently used artemisinin derivatives, namely, artesunate (*oral*), arteether (*i.m.*), and artemether + lumefantrine (*oral*) on haematological parameters. The present investigation was also aimed to study the course of infection in *falciparum*-infected and drug-treated mice to know the efficacy of Artemisinin derivatives based on parasite clearance time (PCT). Thus the aim of our study was to investigate the different hematological changes with *P. falciparum* malaria and to define the possible role of *Plasmodium* species in the pathogenesis related to haematological changes.

The article "A Study on Course of Infection and Haematological Changes in falciparum-Infected in Comparison with Artemisinin(s)-Treated Mice" was retracted in 2014. Reasons: errors in the data; errors in the results or conclusions; concerns about the data; concerns about the results or conclusions.

## 2. Materials and Methods

### 2.1. Animals

C57BL/6J male mice of age of 10-week-old were purchased from National Centre for Laboratory Animal Sciences (N.C.L.A.S), National Institute of Nutrition (NIN), Hyderabad, India, and allowed to acclimatize for 15 days. Animals were fed with standard feed daily and water was given *adlibitum* at room temperature of 24 ± 5°C with 12 hrs. light and dark cycle. The study was conducted in accordance with guidelines in the Guide of the Care and Use of Laboratory Animals [14]. 

### 2.2. Diagnosis, Collection, and Storage of Blood

For the present experiment the species of *P. falciparum* was collected from an infected person from Government General Hospital in Guntur, Andhra Pradesh. Patient is tested with SD BIOLINE Malaria rapid test (P.f/p.v) and blood smear examination by 10 to 15 years experienced microbiologist who confirmed *P. falciparum* with high parasitaemia. At the time of blood collection the patient does not receive any preantimalarial treatment even paracetamol. The blood containing *P. falciparum* was extracted from peripheral vein of hand of the infected individual using 5 mL sterile syringe. Immediately blood was transferred to EDTA vacutainer (BD Franklin, USA); kept in thermocol ice box, and transferred to the laboratory. The obtained antigen was inoculated into the mice within half an hour of collection.

### 2.3. Preparation and Inoculation of Antigen

The collected blood was washed several times in phosphate buffered saline (PBS, pH 7.0) by centrifugation at 1000 rpm/15 min. The washed erythrocytes were suspended in PBS and packed by centrifugation, and supernatant was removed by a pipette. The sediment with *P. falciparum*-infected erythrocytes was diluted with PBS. After obtaining *P. f.* antigen, the parasites were maintained experimentally in three C57BL/6J male mice, and the level of parasitaemia was monitored after the next day of inoculation by smear preparation. After the achievement of high level of parasitaemia (stock blood), blood samples were collected and diluted in normal saline at the ratio of 75% parasitized blood and 25% PBS. The diluted parasitized blood was then inoculated into different experimental mice groups on day “0” via intraperitoneal (*i.p.*) route because malaria parasite penetrates the peritoneal wall into the blood stream within one minute of inoculation. Mice of control group were inoculated with distilled water on day “0” and maintained as control.

The article "A Study on Course of Infection and Haematological Changes in falciparum-Infected in Comparison with Artemisinin(s)-Treated Mice" was retracted in 2014. Reasons: errors in the data; errors in the results or conclusions; concerns about the data; concerns about the results or conclusions.

### 2.4. Drug Administration

A total number of 40 C57BL/6J male mice were distributed into 5 groups, namely, control (CON), infected (INF), drug treated with artesunate (DT AS), drug treated with arteether (DT AE) and drug treated with artemether + lumefantrine (DT AL) of 8 animals each. For all drug-treated groups, therapeutic dosages according to WHO recommendation were administered. Doses were calculated according to the average body weight of the mice (approximately 30 gm/mouse). For monotherapy, artesunate (AS) tablets (Falcigo) from Zydus Cadila Health Care Limited, India, and arteether (AE) (E Mal) from Themis Chemicals Limited, Mumbai, India, were obtained. For combination therapy, artemether + lumefantrine (AL) (Lumerax-20 DT) from Ipca Laboratories Limited, India, was obtained.

- *Artesunate*: through oral gavage in 4 (double divided dose), 2, 2, 2, and 2 mg/kg body weight for five days.
- *Arteether*: intramuscularly in 3 mg/kg body weight for three days.
- *Artemether + Lumefantrine*: through oral gavage in 3.5 mg/kg body weight for three days.

### 2.5. Course of Infection

Course of infection was studied in all the 12-week C57BL/6J experimental mice. Parasitaemia was monitored daily up to day “42” by making peripheral blood smears. Comparison of parasitaemia between infected mice and drug-treated mice revealed the efficacy of each drug used for the study. Thin blood films were made on the prelabelled slide with free flowing whole blood directly from the mouse tail snips after the first drop was wiped off with cotton wool. The blood films were stained with JSB I and JSB II for the detection of malarial parasites and for estimation of parasitaemia. After staining, slides were washed with tap water to remove excess stain and allowed to drain in a vertical position and to air dry. A field was selected where the RBCs are in an evenly distributed monolayer and observed under 100x oil immersion objective. A minimum of 1000 RBCs were counted from 10 fields under microscope, and the number of infected RBCs will be recorded. The percent of parasitaemia was determined by enumerating the number of infected RBCs per total number of RBCs counted (5):

(1) $$\begin{array}{c} \text{parasitaemia}\%=\frac{\text{no}.\;\text{of}\;\text{infected}\;\text{RBCs}}{\text{no}.\;\text{of}\;\text{RBCs}\;\text{counted}}\times 100. \end{array}$$

### 2.6. Evaluation of Responses

Parasite clearance time (PCT) was defined as the time from the start of treatment until first negative blood smear for asexual stages which remained negative for an additional 24 hours. For our study we followed 42-day followup for all treatment groups. Thus PCT was observed in all the experimental groups. 

The article "A Study on Course of Infection and Haematological Changes in falciparum-Infected in Comparison with Artemisinin(s)-Treated Mice" was retracted in 2014. Reasons: errors in the data; errors in the results or conclusions; concerns about the data; concerns about the results or conclusions.

### 2.7. Estimation of Haematological Parameters

At the end of the series of experiments (i.e., after achieving first negative blood smear), 6 animals in all the drug-treated groups were sacrificed using chloroform anaesthesia. Six animals in infected and six animals in control group were sacrificed on day 28. Two animals in all the groups kept for 42 days, and one animal is used to calculate parasitaemia on each day. Blood samples were collected by cardiac puncture into EDTA vacutainer to see the frequency of haematological abnormalities especially anaemia, thrombocytopenia, and reduced blood counts in malaria. Whole blood was immediately analyzed for complete blood picture (CBP), that is, red blood cell (RBC) count, haemoglobin (HGB), hematocrit (HCT), mean cell volume (MCV), mean cell haemoglobin (MCH), mean cell haemoglobin concentration (MCHC), white blood cell (WBC) count, and platelet (PLT) count using the fully automated ABX Pentra 60 + Analyser (Horiba ABX, Montpellier, France). Briefly, 53 *µ*L of blood was aspirated into a needle divided and distributed to the various chambers for sample analysis.

### 2.8. Statistical Analysis

The means, standard deviations of normally distributed data were compared between control versus infected group and infected versus drug-treated groups using Student's *t*-test with MINITAB 11.12.32. Bit statistical package and graphs were drawn from MS Excel 2010. The values were given as mean ± SD and are statistically significant at *t* > 2.306, *P* < 0.05* (significant), *P* < 0.001** (more significant), and *P* < 0.0001*** (highly significant). *P* value more than 0.05 was considered as statistically not significant (NS).

## 3. Results

### 3.1. Observation of *Plasmodium falciparum* Erythrocytic Stages (Asexual Forms)

In the present study,* P. falciparum* erythrocytic stages were developed in the blood of C57BL/6J mouse model after inoculation of 0.3 mL. of *P. f* antigen intramuscularly to the experimental mice. Various stages of parasite are seen in the blood films stained with JSB-I and JSB-II solutions. The blood films were scanned under high power objective (×40) and examined closely under oil immersion objective (×100). The various erythrocytic stages of *P. falciparum* were seen such as trophozoites (immature and mature), schizonts, and gametocyte. Appearance of ring forms at the edge of RBC is the characteristic feature of *Plasmodium falciparum* species (Figure 5).

The erythrocytic stages observed were as follows.

1. *Immature Trophozoite*: undivided nucleated cells with blue-coloured cytoplasm or a ring of cytoplasm within the red cell.
2. *Mature Trophozoite*: compact cytoplasm, enlarged amoeboid shape, and no ring structure.
3. *Schizont*: individual nucleated cell distributed throughout the red cell in a circle.

The article "A Study on Course of Infection and Haematological Changes in falciparum-Infected in Comparison with Artemisinin(s)-Treated Mice" was retracted in 2014. Reasons: errors in the data; errors in the results or conclusions; concerns about the data; concerns about the results or conclusions.

### 3.2. Study of Course of Infection in *Plasmodium falciparum*-Infected Mice

After inoculation of* P. f.* antigen on day “0” into the mice of infected (INF) group, the parasites started developing in the peripheral blood from day “1” onwards and reached to peak level on 11th day with 38% parasitaemia. Then the parasitaemia gradually decreased and completely disappeared by day 28 (Figure 1). 

### 3.3. Effect of Artesunate on *Plasmodium falciparum* in Experimental Mice

After inoculating *P. f.* antigen to mice of DT AS group, parasitic ring stags have appeared on 1st day. Then artesunate drug was administered orally for the next 5 days successively with 2 mg/kg body weight with a double divided dose on the first day. After treating the mice with drug, the peak level of infection was observed on day “3” with 3.5% of parasitaemia only. Then the parasitaemia gradually decreased and disappeared on the 6th day. But the blood smears were examined till the 42nd day and no parasites were observed (Figure 2). The Parasite Clearance Time (PCT) was 144 hours (6 days) with artesunate.

### 3.4. Effect of Arteether on *Plasmodium falciparum* in Experimental Mice

After inoculation of *P. f.* antigen to mice of DT AE group, parasitic ring stags have appeared on the 1st day. Arteether was administered (*i.m.*) on successive 3 days. After Arteether treatment, the peak level of infection was observed on day “2” with 4.2% parasitaemia. Then the parasites were completely disappeared by the 5th day (Figure 3). The Parasite Clearance Time (PCT) was 120 hours (5 days) with arteether. 

### 3.5. Effect of Artemether + Lumefantrine on *Plasmodium falciparum* in Experimental Mice

After giving *P. f.* antigen to the mice in DT AL group, parasitic ring stages have appeared on the 1st day. Then artemether + lumefantrine (artemisinin based combination therapy) was administered orally for the next three days. With the combination therapy, peak level of infection was observed on day “3” with 3.2% parasitemia, and no parasites were observed on day “4” till the 42nd day (Figure 4). The Parasite Clearance Time (PCT) was 96 hours (4 days) with artemether + lumefantrine. 

### 3.6. Changes in Haematological Values of Experimental C57BL/6J Mice due to *Plasmodium falciparum*

Table 1 shows changes in haematological values between control versus infected group. In the infected group the mean value for HGB is 7.93 ± 0.175 (*P* < 0.0001), RBC is 5.9 ± 0.201 (*P* < 0.0001), PCV is 2892 ± 1.46 (*P* < 0.0001), MCV is 81.07 ± 2.19 (<0.0001), MCH is 27.67 ± 1.17 (0.0001), PLT is 516 ± 23.4 (<0.0001), WBC is 6957 ± 102 (<0.0001), neutrophils is 28.3 ± 0.724 (*P* < 0.0001), lymphocytes is 69.70 ± 2.00 (*P* < 0.0001), and eosinophils is 1.0 ± 0.669 (*P* < 0.014). And these values were significantly decreased when compared to the control values (12.85 ± 0.321, 8.0 ± 0.141, 38.67 ± 1.97, 91.48 ± 1.64, 32.33 ± 1.26, 685 ± 20.7, 9080 ± 98.9, 36.15 ± 0.693, 59.85 ± 2.00, and 2.0 ± 0.187), respectively. MCHC (33.17 ± 1.08, *P* > 0.05) and monocytes (1.0 ± 0.190, *P* > 0.05) have not shown significant change in the infected group when compared to control values (34.42 ± 1.12, 1.0 ± 0.228), respectively. 

The article "A Study on Course of Infection and Haematological Changes in falciparum-Infected in Comparison with Artemisinin(s)-Treated Mice" was retracted in 2014. Reasons: errors in the data; errors in the results or conclusions; concerns about the data; concerns about the results or conclusions.

Table 2 shows changes in haematological values in infected (INF) versus artesunate drug-treated (DT AS) group. Significant changes were observed in HGB (*P* < 0.0001), RBC (*P* < 0.0001), PCV (*P* < 0.01), MCV (*P* < 0.01), PLT (*P* < 0.0001), WBC (*P* < 0.001), neutrophils (*P* < 0.0001), lymphocytes (*P* < 0.0001), and eosinophil (*P* < 0.05) in artesunate-treated group when compared with control. MCH (*P* > 0.05), MCHC (*P* > 0.05), and monocytes (*P* > 0.05) did not show statistically significant difference between INF and DT AS groups.

Table 3 shows changes in haematological values in infected (INF) versus arteether drug-treated (DT AE) group. HGB (*P* < 0.0001), RBC (*P* < 0.0001), PCV (*P* < 0.05), PLT (*P* < 0.0001), WBC (*P* < 0.001), neutrophils (*P* < 0.0001), lymphocytes (*P* < 0.0001), and eosinophil (*P* < 0.05) values were significantly increased in DT AE group when compared to INF group. MCV (*P* > 0.05), MCH (*P* > 0.05), MCHC (*P* > 0.05), and monocytes (*P* > 0.05) have not shown significant change in DT AE group when compared to INF group. 

Table 4 shows changes in haematological values in infected (INF) versus artemether + lumefantrine drug-treated (DT AL) group. HGB (*P* < 0.0001), RBC (*P* < 0.0001), PCV (*P* < 0.01), MCV (*P* < 0.001), PLT (*P* < 0.0001), WBC (*P* < 0.001), neutrophils (*P* < 0.0001), lymphocytes (*P* < 0.01), and eosinophil (*P* < 0.05) in artemether + lumefantrine-treated group have significantly increased when compared to the infected group. Insignificant changes were observed for MCH (*P* > 0.05), MCHC (*P* > 0.05), and monocytes (*P* > 0.05) between INF and DT AL groups.

## 4. Discussion

Severe *falciparum* malaria is associated with large parasite burdens. The peripheral blood parasite count is the prognostic indicator that correlates with the total parasite biomass and thus the severity of *falciparum* malaria. Haematological abnormalities are considered a hallmark of malaria and reported to be the most pronounced in *P. falciparum* infection, probably as a result of the higher levels of parasitaemia [15]. This study was conducted to assess and compare the incidence and severity of haematological changes in *falciparum*-infected C57BL/6J mice using an experimental model.

The article "A Study on Course of Infection and Haematological Changes in falciparum-Infected in Comparison with Artemisinin(s)-Treated Mice" was retracted in 2014. Reasons: errors in the data; errors in the results or conclusions; concerns about the data; concerns about the results or conclusions.

In this study we observed that there is a marked reduction in RBC count, WBC count, haemoglobin (HGB), packed cell volume (PCV), mean cell volume (MCV), and platelet counts in *falciparum*-infected mice when compared to control animals. The reduction was more evident in *falciparum *infection. It is thought to result from a combination of haemolysis of parasitized red blood cells, accelerated removal of both parasitized and innocently unparasitized red cells, depressed as well as ineffective erythropoiesis with dyserythropoietic changes, and anaemia of chronic disease [15]. Other factors contributing to anaemia in malaria include decreased red blood cell deformability, splenic phagocytosis, and/or pooling. So they have an increased rate of clearance from the circulation [16]. Malaria parasite within RBCs, ingest and digest haemoglobin more than it needs for its own metabolism. Destruction of RBC following parasitisation cannot account for the degree of anaemia observed during malaria infection, suggesting that the destruction of uninfected RBC (uRBC) is the major cause of haemoglobin (HGB) loss [17].

The low PCV value with a correspondent high density of malaria parasite was suggested to be due to excessive destruction of red blood cells by the malaria parasites. As noted in this study, it was established that the more malaria parasites in the blood circulation cause more destruction of the red blood cells as demonstrated by the low PCV. The low PCV may necessitate the need for blood transfusion which in turn has a high risk of transmitting viral hepatitis, HIV, and other associated risks. The significant reduction in PCV level indicates a relationship between malaria parasite and anaemia [18].

Statistically insignificant changes were observed in MCHC (*P* > 0.05) and monocyte (*P* > 0.05) values in infected mice when compared to control mice. MCHC levels were not significantly changed which is consistent with the earlier reports [19]. In our study we observed that there was a significant reduction in total WBC counts (*P* < 0.0001). Leucopenia appears to be a common finding in both nonimmune patients with *falciparum* malaria and semi-immune children living in malaria-endemic regions [20]. The differential leucocyte count showed normal monocytic, eosinophilic counts and decreased neutrophilic counts. Similarly in the majority of cases, either neutropenia or neutrophilia was reported [20]. Phagocytosis of malaria pigment is by monocyte/macrophages and less frequently by neutrophils [15, 20, 21]. Monocytes and rarely neutrophils contained malaria pigment and in very rare cases, erythrophagocytosis by monocytes was also observed in some studies. Our findings also showed that artemisinin(s) given at the therapeutic doses may not cause neutropenia, which is consistent with prior studies [22, 23].

The article "A Study on Course of Infection and Haematological Changes in falciparum-Infected in Comparison with Artemisinin(s)-Treated Mice" was retracted in 2014. Reasons: errors in the data; errors in the results or conclusions; concerns about the data; concerns about the results or conclusions.

Lymphocytes, particularly T cells, play a major role in immunity to *falciparum* malaria by releasing proinflammatory cytokines. However excessive secretion of proinflammatory cytokines has been shown to contribute to the severity in humans [24–26]. Our study showed that mice infected with *falciparum* had a higher lymphocytic count, and this may represent overstimulation of the proinflammatory pathway. Further studies on the role of lymphocytes are required to determine the significance of our findings.

It is a general consensus that thrombocytopenia is very common in *falciparum* malaria [27, 28] and usually believed that a significant reduction in platelet counts (*P* < 0.0001) than control animals. Thrombocytopenia seems to be due mainly to a reduced platelet life span and splenic pooling. The reduced platelet life span may be caused by binding of malaria antigen onto platelets followed by antibody-mediated phagocytosis [29] or to platelet activation in vivo. Macrophage activation and hyperplasia especially in the spleen may also play a role [30]. The release of platelet contents can activate the coagulation cascade and contributes to decreased inhibitors concentration and consequently further thrombocytopenia [31].

Artemisinin derivatives are most effective against *Plasmodium* parasite (as monotherapies); combination therapies consisting of artemisinin(s) and other antimalarial drugs have been demonstrated to have better parasite clearance and efficacies [32–34]. Antimalarial treatment with artemisinin or one of its derivatives is associated with a more rapid decline in parasitaemia than with other antimalarial drugs [35]. Artemisinins induce a decrease in parasitized RBC deformability. In the presence of heme Fe^++^, these drugs generate carbon centered free radicals that could damage the RBC membrane or cytoskeleton and thereby increase the rigidity of the infected RBC. Artesunate, by acting on young ring forms, attenuated the reduction in deformability parasite, prevented their development to more rigid mature trophozoites, and thereby attenuated the reduction in deformability associated with continued parasite growth. Artesunate induces changes either in the parasite or in the RBC directly and led to increased antigenicity and thus increased opsonization. Terminal half-lives of the orally administered drugs are usually less than 2 h. We observed that once daily administration with artemisinin derivatives provides equivalent cure rates to more frequent administration which is consistent with prior studies [36, 37]. In artesunate group peak of parasitaemia on day 3 with 3.5% and parasites were completely cleared on day 6. First negative blood smear observed on day 6. The peak level of parasitaemia was reduced when compared to AE-treated group (4.2% on day 2). Insignificant changes were observed in MCH (*P* > 0.05), MCHC (*P* > 0.05), and monocytes (*P* > 0.05) for artesunate-treated group.

The article "A Study on Course of Infection and Haematological Changes in falciparum-Infected in Comparison with Artemisinin(s)-Treated Mice" was retracted in 2014. Reasons: errors in the data; errors in the results or conclusions; concerns about the data; concerns about the results or conclusions.

Alpha beta arteether is an ethyl derivative of artemisinin which is an efficient schizonticidal drug in mild malaria. The clinical efficacy of arteether is characterized by an almost immediate onset and rapid reduction in parasitaemia, with complete clearance in most cases within 48 hours. But in our study we observed delayed parasite clearance time in AE-treated groups when compared to previous studies. In arteether group parasites cleared on day 5. We observed positive blood smears for one additional day after the completion of 3-day drug course. The peak level of parasitaemia (4.2% on day 2) was increased when compared to AS-treated group (4 on day 2). Insignificant changes were observed in MCV (*P* > 0.05), MCH (*P* > 0.05), MCHC (*P* > 0.05), and monocytes (*P* > 0.05) for arteether-treated group. No adverse effects were observed on hematological parameters when animals-treated with *α*, β arteether which are consistent with prior studies [38, 39].

AE showed lower efficacy than AL and AS. The levels of efficacy are similar to the findings of the recent studies on ACTs in Africa which revealed that AL has higher efficacy rates when compared to other antimalarials [40–43]. In our study we observed rapid parasite clearance in artemether + lumefantrine-treated group in comparison with artesunate- and arteether-treated animals which are in agreement with previous studies. Our results strongly support that combination therapies have high efficacy rates than monotherapy. Artemisinin(s) can be used alone, but this leads to high rate of recrudescence (return of parasites), and there is a possibility of emergence of resistant strains to the single drug treatment on repeated and inappropriate use and other drugs are required to all parasites and to prevent recrudescence [44]. But in our study no parasite recrudescence was observed in monotherapy and combination therapy. But there is a marked variation in peak level parasitaemia and clearance time. In AL group parasites cleared on day 4. We observed positive blood smears for one additional day after the completion of 3-day drug course. The peak level of parasitaemia (3.2% on day 3) was decreased when compared to AS- (4%) and AE- (4.2%) treated groups. The rate of parasite clearance was used as a measure of the artemisinin pharmacodynamic effect in vivo [35]. Artemisinin resistance is characterized by prolongation in clearance times [18]. There is clear evidence that combinations improve efficacy without increasing toxicity. We found higher efficacy rates when animals were treated with combination (AL) drug than monotherapy. We observed positive blood smears on day 3 for all treatment groups. When compared to AS and AE groups, AL group showed higher efficacy rates by clearing parasites on day 4. Insignificant changes were observed in MCHC (*P* > 0.05) 0 and monocytes (*P* > 0.05) for artemether + lumefantrine-treated group.

The article "A Study on Course of Infection and Haematological Changes in falciparum-Infected in Comparison with Artemisinin(s)-Treated Mice" was retracted in 2014. Reasons: errors in the data; errors in the results or conclusions; concerns about the data; concerns about the results or conclusions.

## 5. Conclusion 

Considering the higher efficacy rates of artemether +lumefantrine (AL) as compared with artesunate (AS) and arteether (AE), we conclude that AL is clinically more effective than AS and AE. No adverse effects were observed on haematological parameters when animals were treated with artemisinin derivatives. Artemisinin resistance is characterized by prolongation in clearance times which we observed in the present study. The result of *falciparum* positive blood smear in all treatment groups on day 3 (72 h) was a good predictor for treatment failure and considered as a simple screening measure for artemisinin resistance. 

## Figures and Tables

**Figure 1:** Course of infection to *Plasmodium falciparum* in experimental C57BL/6J mice.

**Figure 2:** Effect of artesunate on *Plasmodium falciparum* in experimental C57BL/6J mice.

**Figure 3:** Effect of arteether on *Plasmodium falciparum* in experimental C57BL/6J mice.

**Figure 4:** Effect of artemether + lumefantrine on *Plasmodium falciparum* in experimental C57BL/6J mice.

**Figure 5:** Developmental stages of *Plasmodium falciparum* in C57BL/6J mice blood. ((a) and (b)) Ring form or early trophozoite. ((c) and (d)-A) Developing trophozoite. (d)-B Early schizont. (e) Mature trophozoite showing clumped pigment. (f) Trophozoite.

**Table 1:** Changes in haematological values between control versus infected mice.

Parameter	Experimental group (*N* = 6)		*t* value	*P* value
	Control (CON)	Infected (INF)		
	(Day 28)	(Day 28)		
HGB (g/dL)	12.85 ± 0.321	7.93 ± 0.175	32.94	<0.0001***
RBC (10^6^/mm^3^)	8.0 ± 0.141	5.90 ± 0.201	20.84	<0.0001***
PCV (%)	38.67 ± 1.97	28.92 ± 1.46	9.74	<0.0001***
MCV (fL)	91.48 ± 1.64	81.07 ± 2.19	9.34	<0.0001***
MCH (pg)	32.33 ± 1.26	27.67 ± 1.17	6.65	<0.0001***
MCHC (g/dL)	34.42 ± 1.12	33.17 ± 1.08	1.96	>0.05^ NS^
PLT (10^3^/mm^3^)	685 ± 20.7	516.7 ± 23.4	13.19	<0.0001***
WBC (cells/mm^3^)	9080 ± 98.9	6957 ± 102	36.61	<0.0001***
Neutrophils (%)	36.15 ± 0.693	28.3 ± 0.724	21.65	<0.0001***
Lymphocytes (%)	59.85 ± 2.00	69.70 ± 2.00	8.53	<0.0001***
Monocytes (%)	1.0 ± 0.228	1.0 ± 0.117	0.00	>0.05^ NS^
Eosinophils (%)	2.0 ± 0.187	1.0 ± 0.669	3.70	<0.05*

The values are given as mean ± SD are statistically significant at *t* > 2.306, *P* < 0.05*, *P* < 0.001**, and *P* < 0.0001***; not significant at *P* > 0.05; HGB: hemoglobin; RBC: red blood cells; PCV: packed cell volume; MCV: mean cell volume; MCH: mean cell hemoglobin; MCHC: mean cell hemoglobin concentration; PLT: platelets; WBC: white blood cells.

The article "A Study on Course of Infection and Haematological Changes in falciparum-Infected in Comparison with Artemisinin(s)-Treated Mice" was retracted in 2014. Reasons: errors in the data; errors in the results or conclusions; concerns about the data; concerns about the results or conclusions.

**Table 2:** Changes in haematological values between infected versus artesunate drug-treated mice.

Parameter	Experimental group (*N* = 6)			
	(at the end of the experiment after parasite clearance)		*t* value	*P* value
	Infected (INF)	Drug-treated artesunate (DT AS)		
HGB (g/dL)	7.93 ± 0.175	11.20 ± 0.846	9.28	<0.001**
RBC (10^6^/mm^3^)	5.90 ± 0.201	7.95 ± 0.0894	22.73	<0.0001***
PCV (%)	28.92 ± 1.46	33.67 ± 2.94	3.54	<0.05*
MCV (fL)	81.07 ± 2.19	86.83 ± 3.19	3.65	<0.05*
MCH (pg)	27.67 ± 1.17	28.43 ± 0.625	1.42	>0.05^ NS^
MCHC (g/dL)	33.17 ± 1.08	32.75 ± 1.73	0.50	>0.05^ NS^
PLT (10^3^/mm^3^)	516.7 ± 23.4	675 ± 11.0	15.02	<0.0001***
WBC (cells/mm^3^)	6957 ± 102	8700 ± 522	8.04	<0.001**
Neutrophils (%)	28.3 ± 0.724	40 ± 0.754	27.43	<0.0001***
Lymphocytes (%)	69.70 ± 2.00	57.67 ± 2.80	8.56	<0.0001***
Monocytes (%)	1.0 ± 0.117	1.0 ± 0.126	0.00	>0.05^NS^
Eosinophils (%)	1.0 ± 0.669	2.0 ± 0.518	2.69	<0.05*

The values are given as mean ± SD are statistically significant at *t* > 2.306, *P* < 0.05*, *P* < 0.001**, and *P* < 0.0001***; not significant at *P* > 0.05; HGB: hemoglobin; RBC: red blood cells; PCV: packed cell volume; MCV: mean cell volume; MCH: mean cell hemoglobin; MCHC: mean cell hemoglobin concentration; PLT: platelets; WBC: white blood cells.

**Table 3:** Changes in haematological values between infected versus arteether drug-treated mice.

Parameter	Experimental group (*N* = 6)			
	(at the end of the experiment after parasite clearance)		*t* value	*P* value
	Infected (INF)	Drug-treated arteether (DT AE)		
HGB (g/dL)	7.93 ± 0.175	11.08 ± 0.770	29.53	<0.0001***
RBC (10^6^/mm^3^)	5.90 ± 0.201	7.73 ± 0.154	17.66	<0.0001***
PCV (%)	28.92 ± 1.46	31.67 ± 1.86	2.84	<0.05*
MCV (fL)	81.07 ± 2.19	86.17 ± 5.49	2.11	>0.05^NS^
MCH (pg)	27.67 ± 1.17	27.6 ± 1.23	0.10	>0.05^NS^
MCHC (g/dL)	33.17 ± 1.08	33.35 ± 0.985	0.30	>0.05^NS^
PLT (10^3^/mm^3^)	516.7 ± 23.4	650 ± 22.8	10.00	<0.0001***
WBC (cells/mm^3^)	6957 ± 102	8983 ± 475	10.22	<0.001***
Neutrophils (%)	28.3 ± 0.724	37.01 ± 0.708	21.08	<0.0001***
Lymphocytes (%)	69.70 ± 2.00	60.67 ± 1.63	8.57	<0.0001***
Monocytes (%)	1.0 ± 0.117	1.0 ± 0.210	8.57	>0.05^NS^
Eosinophils (%)	1.0 ± 0.669	2.0 ± 0.729	8.57	<0.05*

The values are given as mean ± SD are statistically significant at *t* > 2.306, *P* < 0.05*, *P* < 0.001**, and *P* < 0.0001***; not significant at *P* > 0.05; HGB: hemoglobin; RBC: red blood cells; PCV: packed cell volume; MCV: mean cell volume; MCH: mean cell hemoglobin; MCHC: mean cell hemoglobin concentration; PLT: platelets; WBC: white blood cells.

The article "A Study on Course of Infection and Haematological Changes in falciparum-Infected in Comparison with Artemisinin(s)-Treated Mice" was retracted in 2014. Reasons: errors in the data; errors in the results or conclusions; concerns about the data; concerns about the results or conclusions.

**Table 4:** Changes in haematological values between infected versus artemether-lumefantrine drug-treated mice.

Parameter	Experimental group (*N* = 6)			
	(at the end of the experiment)		*t* value	*P* value
	Infected (INF)	Drug-treated artemether-lumefantrine (DT AL)		
HGB (g/dL)	7.93 ± 0.175	11.08 ± 0.770	9.77	<0.001**
RBC (10^6^/mm^3^)	5.90 ± 0.201	7.78 ± 0.317	12.23	<0.0001***
PCV (%)	28.92 ± 1.46	33.67 ± 2.94	3.54	<0.05*
MCV (fL)	81.07 ± 2.19	87.0 ± 1.79	5.14	<0.001**
MCH (pg)	27.67 ± 1.17	28.7 ± 1.16	1.54	>0.05^NS^
MCHC (g/dL)	33.17 ± 1.08	33.33 ± 1.34	1.54	>0.05^NS^
PLT (10^3^/mm^3^)	516.7 ± 23.4	680 ± 11.4	15.38	<0.0001***
WBC (cells/mm^3^)	6957 ± 102	8033 ± 378	6.74	<0.001**
Neutrophils (%)	28.3 ± 0.724	41.00 ± 1.41	19.58	<0.0001***
Lymphocytes (%)	69.70 ± 2.00	58.33 ± 4.55	5.61	<0.001**
Monocytes (%)	1.0 ± 0.117	1.0 ± 0.297	0.00	>0.05^NS^
Eosinophils (%)	1.0 ± 0.669	2.0 ± 0.566	0.00	<0.05*

The values are given as mean ± SD are statistically significant at *t* > 2.306, *P* < 0.05*, *P* < 0.001**, and *P* < 0.0001***; not significant at *P* > 0.05; HGB: hemoglobin; RBC: red blood cells; PCV: packed cell volume; MCV: mean cell volume; MCH: mean cell hemoglobin; MCHC: mean cell hemoglobin concentration; PLT: platelets; WBC: white blood cells.
